RETRACTED

# Influence of Continuous Nursing Intervention on Treatment Compliance of Patients with Depression

**DOI:** 10.1155/2022/7080678

**Published:** 2022-09-23

**Authors:** Yanfang He, Jie He, Xueyuan Hou

**Affiliations:** Department of Psychiatry, Huai'an No. 3 People's Hospital, Huai'an 223001, Jiangsu, China

## Abstract

**Objective:**

This study mainly discusses the influence of the continuous nursing intervention on the treatment compliance of patients with depression.

**Methods:**

The clinical data of 120 patients with depression admitted to our hospital were collected by retrospective analysis. According to the different implementation of nursing methods, patients were subordinated to the conventional group (*n* = 48, conventional nursing) and the continuous group (*n* = 72, continuous nursing). The treatment compliance, depression degree, quality of life, nursing satisfaction, Insight and Treatment Attitude Questionnaire (ITAQ), and recurrence rate of patients in the two groups were compared.

**Results:**

The continuous group had a higher treatment compliance rate, slighter depression, higher physiological function, psychological function, social function, environmental adaptability, total quality of life, nursing satisfaction, and ITAQ score, and lower recurrence rate, with statistically significant differences (*P* < 0.05).

**Conclusion:**

The implementation of continuous nursing intervention for patients with depression could enhance their treatment compliance and relieve depressive symptoms; improve the quality of life and self-awareness; reduce the risk of relapse; and improve nursing satisfaction.

## 1. Introduction 

Depression is a common mental disorder in psychiatry. In China, the annual incidence rate is 3%–5%, and the annual recurrence rate is as high as 37.51%, which has become the second major disease in the world [1]. Typical clinical manifestations of the disease include willful activity disorder, thinking delay, and persistent depression, etc., and somatic symptoms of varying degrees may occur in severe cases [2]. Depression patients were often accompanied by emotional instability, if the patient's condition is more serious, it is easy to make harmful social behavior. If the patient does not receive effective treatment in time, there will be suicidal thoughts and even suicidal behavior, which will threaten the life, health, and safety of the patient. As depression is a chronic disease, the clinical treatment of depression, mainly, adopts long-term standardized use of antidepressants, which can effectively control the patient's condition [3]. However, due to the long treatment cycle of depression, it is easy to lead to poor treatment compliance in patients, which will adversely affect the treatment. Therefore, on the basis of strict standard treatment, it is of great significance to cooperate with effective nursing measures. Conventional nursing measures have a single form and insufficient strength to improve patients' treatment compliance, which make it difficult to ensure that patients get good treatment benefits. Therefore, it is necessary to explore a new, effective, and adjuvant nursing intervention. Continuous care is a newly introduced nursing model in recent years. This nursing service is not limited by the discharge of patients but can be extended to the community and family as patients return to society [4]. Continuous nursing has been reported in many departments and achieved good results [5]. However, there are few reports on the application of this nursing model to patients with depression. Therefore, this study adopted the retrospective analysis method to collect clinical data of 120 patients with depression admitted to our hospital, aiming to analyze the impact of continuous nursing intervention on the treatment compliance of patients with depression in order to provide new guidance for the adjuvant treatment and clinical nursing program of depression so that patients could benefit more. It was found that this kind of intervention could enhance treatment compliance and relieve depressive symptoms, improve the quality of life and self-awareness, reduce the risk of recurrence, and improve nursing satisfaction. The results were reported as follows:

RETRACTED

## 2. Materials and Methods

### 2.1. Data Sources

Retrospective analysis is an observational study. A retrospective study is a method of looking back to the past with the results of the present. Clinical data of patients with depression admitted to our hospital from March 2019 to February 2022 were collected by retrospective analysis. The patients must have the following conditions: (1) after comprehensive clinical examination, it met the clinical diagnostic criteria of Diagnostic and Statistical Manual 4th Edition (DSM-?) depression [6]; (2) initial; (3) no serious suicidal tendency; (4) lack of clinical data. The patients cannot have the following conditions: (1) complicated with serious heart, liver, kidney, and other important organ diseases; (2) unclear consciousness; (3) communication barriers; (4) women in pregnancy or lactation. One hundred and twenty patients were selected for analysis, including 73 male cases and 49 female cases. Their ages were (45.72 ± 5.86) years, the courses of disease were (1.50 ± 0.49) years, and the education levels were (9.36 ± 2.34) years. Patients were subordinated to the conventional group (*n* = 48) and the continuous group (*n* = 72) according to the different nursing delivery styles. A comparison of baseline data between the conventional group and the continuous group showed no statistically significant difference (*P* > 0.05), indicating comparability. The baseline data of the conventional group and the continuous group are shown in Table 1, and the steps of this study were shown in Figure 1.

RETRACTED

### 2.2. Nursing Methods

Patients in the conventional group received the conventional nursing intervention after discharge. Specific methods: (1) the nursing staff gave routine discharge guidance to patients and distributed health education manuals related to depression. (2) Nursing staff conducted propaganda, education, and guidance to patients according to the discharge doctor's advice in discharge records, including relevant matters needing attention after discharge, the use of drugs after discharge, follow-up time, and other information. (3) The nursing staff carried out conventional follow-up for the patients.

Patients in the continuous group received continuous nursing intervention on the basis of conventional nursing after discharge. Before discharge, the nurse in charge sets up continuous nursing files for each patient. The basic information of the patients was recorded, including name, gender, age, occupation, education level, home phone number, the physician in charge, the nurse in charge, time of admission, and discharge, admission and discharge diagnosis, the treatment plan during hospitalization, treatment plan for discharge, and scores of depression-related scales. Specific methods: nursing staff to patients with continuous telephone follow-up and reasonable healthy guidance. (1) Staffing: the charge nurse during the patient's hospitalization should be selected to undertake follow-up tasks. The charge nurse should have solid professional knowledge of depression and good communication skills and experience. (2) Close follow-up: patients were followed up by telephone twice a month for the first three months after discharge and once a month thereafter, with each follow-up lasting about 30 minutes. Follow-up contents: comprehensive understanding of patients' psychological and emotional state, diet, sleep, and medication status; inquire carefully about the patient's psychological and therapeutic care needs; explain and guide the problems of patients during medication; psychological counseling and life guidance for patients with emotional instability; conduct medication compliance guidance and supervision; nursing staff recorded each follow-up in detail to provide reference for the next follow-up.

### 2.3. Observation Indicators and Evaluation Criteria

#### 2.3.1. Treatment Compliance [7]

It includes noncompliance, partial compliance, and full compliance. Noncompliance: patients did not cooperate with medical staff and did not take medication for treatment. Partial compliance: patients took medication under the supervision of medical staff or passively; full compliance: patients actively cooperated with medical staff to take medicine.

RETRACTED

#### 2.3.2. Depression Degree

The degree of depression of patients was assessed by the Self-rating Depression Scale (SDS) [8]. The scale contained 20 items reflecting subjective feelings of depression, and each item was divided into four grades according to the frequency of symptom occurrence, among which 10 items were positive scores (score 1, 2, 3, 4) and 10 items were negative scores (score 4, 3, 2, 1). The result was that the total rough score (*X*) was obtained by adding the scores of the 20 items, and the standard score (*Y*) was obtained by multiplying the rough score by 1.25 and rounding it up. 53–62 were classified as mild depression, 63–72 as moderate depression, and 73 or more as severe depression.

#### 2.3.3. Quality of Life

It was evaluated by the Quality of Life Scale Brief Version (QOL-BREF) [9], including 24 items in 4 dimensions, namely psychological function (6 items), physiological function (7 items), environmental adaptability (8 items), and social function (3 items). Cronbach's *α* coefficient of each dimension was greater than 0.70. The Likert level 5 scoring method was adopted, and the score of each dimension was 1 (completely affected)–5 (not affected), with a total score of 120 the higher the score, the better the quality of life.

#### 2.3.4. Nursing Satisfaction

Patients filled in the nursing satisfaction questionnaire made by our hospital, including dissatisfaction (≤49 points), general satisfaction (50–69 points), satisfaction (70–89 points), and great satisfaction (≥90 points). Degree of satisfaction = (satisfaction + great satisfaction) number of cases/total number of cases × 100%.

The Insight and Treatment Attitude Questionnaire (ITAQ) [10] was scored at discharge, 6 months after discharge, and 12 months after discharge. The questionnaire included 11 items. The scores of each item were 0 (no self-awareness), 1 (partial self-awareness), and 2 (full self-awareness).

The recurrence rate was assessed by the Hamilton Depression Scale (HAMD) [11] at 6 months and 12 months after discharge. The recurrence criterion was the occurrence of significant depressive symptoms with a HAMD score of >20.

### 2.4. Statistical Methods

The SPSS 20.0 software was applied to analyze the data, and the quantitative data was expressed as ($\bar{x}\pm s$). The *t* test was performed for compariso_n_ between the two groups, and repeated measure ANOVA was used for comparison of data at different time points between groups. Qualitative data were expressed by *n* (%), and the chi-square test was performed. When 1≤ theoretical frequency <5, the chi-square value should be corrected, and when the theoretical frequency <1, exact probability method was used to calculate. *P* < 0.05 was considered statistically significant.

RETRACTED

## 3. Results

### 3.1. Treatment Compliance Was Higher in the Continuous Group

Compared with conventional group, the treatment compliance rate of continuous group was higher (*P* < 0.05), as shown in Table 2.

### 3.2. Continuous Group Had Slighter Depression

The depression degree of the continuous group was slighter (*P* < 0.05), as shown in Table 3.

### 3.3. The Survival Quality of the Continuous Group Group Was Higher

Compared with the conventional group, the physiological function, psychological function, social function, environmental adaptability, and total quality of life of the continuous group were higher (*P* < 0.05), as shown in Table 4.

### 3.4. Continuous Group Had Higher Nursing Satisfaction

The nursing satisfaction of the continuation group was 94.44%, higher than the control group's 64.58% (*P* < 0.05), as shown in Table 5.

### 3.5. ITAQ

Compared with the conventional group, the ITAQ score in the continuous group was higher, and the difference was statistically significant (inter-group effect: *F* = 25.740, *P* < 0.001). ITAQ scores in both groups tended to increase with time (time effect: *F* = 38.580, *P* < 0.001). There was an interaction effect between groups and time (interaction effect: *F* = 9.378, *P* < 0.001), as shown in Table 6.

### 3.6. Recurrence Rate

In continuous group, 3 cases recurred within 6 months after discharge, and 6 cases recurred 1 year after discharge; a total of 9 cases (12.50%) recurred. In conventional group, 6 cases recurred within 6 months after discharge, and 16 cases recurred 1 year after discharge, 22 cases recurred (45.83%). The recurrence rate in the continuous group was lower (*χ*^2^ = 15.986, *P* < 0.001).

## 4. Discussion

Depression is a clinical chronic disease, and its onset is affected by the patient's own behavior, psychological quality, social environment, and other factors. The incidence of the disease is high and the treatment cycle is long. Due to the influence of the disease, the depression of patients is aggravated, the medication compliance is low, and the probability of recurrence is increased, which poses a great threat to their life and health. It is of great significance to improve medication compliance and regularity of patients with depression [12]. At present, medication compliance of patients with depression is one of the hot spots in clinical research. Nursing staff and patient contact frequency is higher, so they can systematically understand the actual condition of patients and basic situation. Therefore, on the basis of the establishment of depression a treatment plan supplemented by high-quality nursing mode, it is conducive to patients' better cooperation with the treatment so as to effectively improve the degree of depression and reduce the probability of recurrence.

RETRACTED

This study found that the continuous group had a higher treatment compliance rate (100.00% vs. 81.25%), slighter depression, higher physiological function, psychological function, social function, environmental adaptability, total quality of life, and nursing satisfaction (94.44% vs. 64.58%). It indicated that compared with conventional nursing, continuous nursing could significantly improve patients' treatment compliance, reduce depression, and improve quality of life and nursing satisfaction. The implementation of continuous nursing intervention enabled patients to maintain exchanges and communication with nursing staff, form a good nurse-patient relationship, and improve the feasibility of out-of-hospital nursing intervention without being limited by region and time after discharge. The mutual trust and good nurse-patient relationship between nurses and patients helped patients to understand the health knowledge related to depression so that patients actively cooperated with medical staff for treatment. In addition, nurses informed patients of the pharmacological effects of antidepressants, which was conducive to enhancing patients' awareness of the drugs, and informed patients to adhere to the medication. They also told the patient's family to strictly monitor the patient to take medicine correctly and urged the patient to take medicine on time and in accordance with the amount. These measures were conducive to promoting patients' active cooperation with treatment and improving treatment compliance, which was consistent with previous research results [13]. Patients' treatment compliance could be improved, and they could take antidepressants on time, in regular quantity, and in accordance with the doctor's advice, so that the drugs could play a full role in patients, which could effectively help patients fight depression symptoms and reduce the degree of depression of patients [14]. Depression symptoms of patients were well improved, and their physical, psychological, social, and environmental adaptability were naturally enhanced, so their overall quality of life was improved, which was similar to the results of relevant studies [12]. On the one hand, the patient's treatment compliance was significantly improved, the degree of depression was reduced, and the condition improved. On the other hand, in the process of continuous nursing intervention, nursing staff master the emotional changes and personality characteristics of patients and implemented the corresponding nursing intervention according to the actual condition of the patients. The nurses provided patients with high quality, high efficiency, and good nursing service in two aspects of treatment effect and the relationship between nurses and patients. This made the patients realize the professionalism of the nursing staff and their nursing work so that patients were treated with a positive attitude toward nursing work. So it could improve relationships between nurses and patients and make patient's nursing job satisfaction increase [4].

RETRACTED

According to the results of this study, the continuous group had higher ITAQ score (intergroup effect: *F* = 25.740, time effect: *F* = 38.580, interaction effect: *F* = 9.378) and lower recurrence rate (12.50% vs. 45.83%, 2 = 15.986). This suggests that continuous nursing intervention could improve self-awareness and reduce the recurrence rate of patients with depression. The results of this study suggested that continuity of care from hospital to home was a very effective means to improve the efficacy and prognosis of depression. Because of the importance of continuous nursing to the curative effect and prognosis of disease, the content and mode of continuous nursing intervention have always been a hot topic of nursing research at home and abroad. In the case of underdeveloped community medical services in China, how to ensure that patients can still get adequate nursing and treatment in the family after discharge and how to make nursing treatment in the family become the continuation of hospital nursing treatment is worth studying. According to foreign research reports, continuous nursing includes three core elements, namely, continuity of information; continuity of management; and continuity of relationship [15]. In the process of implementing of continuous nursing in this study, the nursing staff established continuous nursing archives for patients. The archives were not only a detailed record of the patient's personal information and health information but also a timely recording of patient follow-up and feedback material content, highlighting the continuation of information, which was conducive to fully grasping the treatment of the patients and nursing assessment. Nursing practiced the regularity of follow-up after discharge from the hospital, giving patients during patients' psychological counseling, guidance, and supervision of the life. This made the patient can continue to get the corresponding nursing after discharge. This was the continuation of nursing management. It prolonged the auxiliary time during nursing care in the treatment of depression and made depression against treatment carry out more smoothly. During the patient's hospitalization, the nurse in charge of the patient follow-up work fully understood the patient's depression treatment status, which helped to establish a long-term relationship of mutual trust between nurses and patients. This was the continuation of the relationship and was conducive to improving the patient's confidence in cure, so that they take the initiative to accept and cooperate with treatment, so as to reduce recurrence [16]. Continuous nursing was a new and effective nursing intervention. The nursing service was not restricted by the discharge of patients and could be extended to the community and family with the return of patients to society. This nursing method was more diversified than the conventional nursing measures, and it could improve the treatment compliance of patients with greater intensity, so that patients could obtain better treatment benefits.

RETRACTED

## 5. Strengths and Limitations

In this study, the retrospective analysis method was adopted to collect relevant clinical data from patients with initial depression, and conventional nursing was used as the control to observe the influence of continuous nursing on the treatment compliance, depression degree, and recurrence of patients with depression after discharge, which had a certain scientific nature. However, the dataset for the retrospective study were from the past clinical database, and there was a lack of randomized controlled trials, so the study lacked rigor. In addition, due to the small number of cases in this single-center study, the results of the study may be biased. Therefore, future research directions should also shift to prospective control studies and multicenter studies to enhance the reliability of the results of this study.

## 6. Conclusions

The implementation of continuous nursing intervention for patients with depression could enhance their treatment compliance and relieve depressive symptoms, improve the quality of life and self-awareness, reduce the risk of relapse, and improve nursing satisfaction, which is worthy of promotion and application.

## Figures and Tables

**Figure 1:** The steps of this study.

**Table 1:** The baseline data of the conventional group and the continuous group.

Group	Conventional group (*n* = 48)	Continuous group (*n* = 72)	*χ* ^2^/*t*	*P*
*Gender* [*n* (%)]			0.052	0.820
Male	29 (60.42)	42 (58.33)		
Female	19 (39.58)	30 (41.67)		
Age ($\bar{x}\pm s$, year)	45.26 ± 6.13	46.17 ± 5.58	0.841	0.402
Course of disease ($\bar{x}\pm s$, year)	1.52 ± 0.43	1.48 ± 0.55	0.425	0.672
Educational level ($\bar{x}\pm s$, year)	9.13 ± 2.52	9.58 ± 2.15	1.048	0.297

*Compliance* [*n* (%)]			1.182	0.554
Noncompliance	9 (18.75)	9 (12.50)		
Partial compliance	17 (35.42)	31 (43.06)		
Full compliance	22 (45.83)	32 (44.44)		

*Depression degree* [*n* (%)]			4.018	0.134
Mild depression	24 (50.00)	46 (63.89)		
Moderate depression	18 (37.50)	15 (20.83)		
Severe depression	6 (12.50)	11 (15.28)		

RETRACTED

**Table 2:** Comparison of treatment compliance [*n*(%)].

Group	Noncompliance	Partial compliance	Full compliance	Treatment compliance rate
Conventional group(*n* = 48)	9(18.75)	13(27.08)	26(54.17)	39(81.25)
Continuous group(*n* = 72)	0(0.00)	7(9.72)	65(90.28)	72(100.00)

*χ* ^2^	23.947			17.605
*P*	<0.001			<0.001

**Table 3:** Comparison of depression degree [*n*(%)].

Group	No depression	Mild depression	Moderate depression	Severe depression
Conventional group (*n* = 48)	18(37.50)	14(29.17)	13(27.08)	3(6.25)
Continuous group (*n* = 72)	34(47.22)	30(41.67)	8(11.11)	0(0.00)

*χ* ^2^	9.845			
*P*	0.013			

**Table 4:** Comparison of QOL-BREF ($\bar{x}\pm s$, point).

Group	Physiological function	Psychological function	Social function	Environmental adaptability	Total quality of life
Conventional group (*n* = 48)	2.26 ± 0.29	2.03 ± 0.19	3.35 ± 0.38	3.10 ± 0.41	11.24 ± 2.21
Continuous group (*n* = 72)	5.17 ± 0.62	3.96 ± 0.52	5.71 ± 0.52	5.33 ± 0.76	23.55 ± 3.26
*T*	30.350	24.610	26.990	18.590	22.880
*P*	<0.001	<0.001	<0.001	<0.001	<0.001

**Table 5:** Comparison of nursing satisfaction [*n*(%)].

Group	Dissatisfaction	General satisfaction	Satisfaction	Great satisfaction	Degree of satisfaction
Conventional group (*n* = 48)	6(12.50)	11(22.92)	17(35.42)	14(29.17)	31(64.58)
Continuous group (*n* = 72)	0(0.00)	4(5.56)	12(16.67)	56(77.78)	68(94.44)

*χ* ^2^	15.779				32.002
*P*	<0.001				<0.001

**Table 6:** Comparison of ITAQ ($\bar{x}\pm s$, point).

Time	Conventional group (*n* = 48)	Continuous group (*n* = 72)	*t*	*P*
At discharge	15.36 ± 4.16	15.41 ± 3.38	0.072	0.942
6 months after discharge	10.83 ± 4.58	14.89 ± 5.22	4.380	<0.001
12 months after discharge	9.15 ± 3.72	13.62 ± 4.26	5.918	<0.001

## Data Availability

The data used for this study are available from the corresponding author upon request.
